The article "Traditional Chinese medicine intervention for autism spectrum disorders: A protocol for systematic review and network meta-analysis" was retracted in 2022. Reason: concerns about the citations.

# Traditional Chinese medicine intervention for autism spectrum disorders: A protocol for systematic review and network meta-analysis

**DOI:** 10.1097/MD.0000000000028957

**Published:** 2022-03-04

**Authors:** Xiang Feng, Keshang Li, Quanrui Jiang, Yuxing Zhang, Zhichao Gong, Hui Zhi, Jun Yu, Wu Li, Jiangshan Li

**Affiliations:** a School of Acupuncture-Moxibustion and Tuina, Hunan University of Chinese Medicine, Changsha, Hunan, China; b College of Acupuncture and Orthopedics, Hubei University of Chinese Medicine, Wuhan, Hubei, China; c The First Affiliated Hospital of Hunan University of Chinese Medicine, Changsha, Hunan, China.

**Keywords:** autism spectrum disorders, network meta-analysis, protocol, systematic review, Traditional Chinese medicine

## Abstract

**Background:**

Autism spectrum disorder (ASD) is a neurodevelopmental disorder characterized by impairments in social communication, social interaction, and restrictive or repetitive behaviors. Traditional Chinese medicine (TCM) has been used in the clinical management of ASD, especially in mainland China, where studies have shown promising efficacy. However, this remains to be further explored and clarified. Therefore, the purpose of this study was to evaluate the effectiveness and safety of conventional treatment-based TCM interventions for ASD.

**Method:**

The study will be conducted from January 2022, and the following electronic databases will be searched: China Biological Medicine Database, Chinese Scientific Journals Database, Wan Fang database, and China National Knowledge Infrastructure, the Cochrane Library, Web of Science, PubMed, and EMBASE Database. Only randomized controlled trials of TCM interventions for ASD will be included. The Autism Diagnostic Observation Scale, Autism Diagnostic Interview-Revised, and Childhood Autism Rating Scale will be the primary outcome indicators. The methodological quality of this Bayesian-based network meta-analysis will be performed using the “Risk of Bias” tool. Stata 14.0 and WinBUGS 1.4.3 will be used to analyze the data. In addition, assessment of heterogeneity, inconsistency, subgroups, sensitivity, and publication bias will be conducted using the Cochrane Collaboration's tools.

**Results:**

The results of this study will be submitted to a peer-reviewed journal for publication.

**Conclusion:**

This study will help patients recover better, provide clinical evidence for practitioners, and promote the use of TCM in ASD interventions.

## 1 Introduction

Autism spectrum disorder (ASD) is a pervasive neurodevelopmental disability, and the DSM-5 (Diagnostic and Statistical Manual of Mental Disorders, fifth edition) specifies its main core symptoms as impairments in social communication, social interaction, and restrictive or repetitive behaviors.^[1]^ In addition to the two core symptoms, individuals with ASD have some impairments in cognitive functioning and affective behavior.^[2]^ In recent years, the prevalence of autism has increased gradually, and the Centers for Diseases and Control Prevention released the most recent data on the prevalence of autism at the end of 2021, showing that 1 in 44 children are diagnosed with ASD.^[3]^ The cause of ASD has not been identified but is now widely believed to be the result of the interaction between environmental and genetic factors.^[4]^ As research has progressed, rare variants in genes as well as common genetic variants with small effects have been shown to increase the risk of developing ASD.^[5]^

Children with ASD have difficulties in social integration, and some of the core symptoms remain for the rest of their life, requiring long-term rehabilitation. *The Lancet* pointed out that patients with severe ASD currently account for approximately 30% of all ASD patients and that they are in need of more treatment and rehabilitation opportunities.^[6]^ The high cost of rehabilitation and medical expenses puts a heavy burden on society and ASD families.

The article "Traditional Chinese medicine intervention for autism spectrum disorders: A protocol for systematic review and network meta-analysis" was retracted in 2022. Reason: concerns about the citations.

There is no specific treatment for the rehabilitation of ASD, but the main focus of current treatments is on behavioral interventions and physical therapy.^[7]^ Applied Behavior Analysis is a behavioral training model that uses a stimulus-response-reinforcement approach with the goal of developing socially adaptive behaviors, reducing problematic behaviors, and emphasizing parental involvement.^[8]^ Physiotherapy includes transcranial magnetic stimulation, which is often preferred, because of its painlessness and low side effects, to reduce repetitive behaviors and sensitivity to the environment in patients.^[9]^ In contrast, pharmacological treatment is not currently a common intervention, but it has a certain alleviating effect on some ASD symptoms.^[10]^ All of the above treatments have contributed to the recovery of children with ASD.

Traditional Chinese medicine (TCM) has been guarding the health of the Chinese people for thousands of years and has been used to treat diseases through clinical practice using herbal medicines in formulas or external treatments, such as acupuncture, moxibustion, Tuina, and Guasha. However, because of historical reasons, there is a lack of evidence of the effectiveness of TCM, as the use of modern scientific means to continue and standardize research on TCM is relatively recent.

The treatment of ASD by TCM has gradually diversified in the last years, and research progress has been made. In our study, a Bayesian network meta-analysis will be performed to compare the efficacy and safety of different TCM interventions for ASD and to find the optimal treatment combination. This will be the first attempt of its kind in this field.

The article "Traditional Chinese medicine intervention for autism spectrum disorders: A protocol for systematic review and network meta-analysis" was retracted in 2022. Reason: concerns about the citations.

## 2 Methods

### 2.1 Study registration

This study was registered on INPLASY (International Platform of Registered Systematic Review and Meta-analysis Protocols) on January 31, 2022, under number INPLASY202210137. It was updated on February 9, 2022, for consistency with the content of this paper. Any changes in this protocol will be updated in detail.

### 2.2 Ethics

This study only analyzed textual data and did not involve studies with animal or human samples; therefore, no ethical approval was required.

### 2.3 Selection criteria

#### 2.3.1 Types of studies

The study will focus on all complete randomized controlled trials of TCM interventions in ASD, and subjects from any ethnic background will be included in the study. However, language will be limited to studies published in English or Chinese only, and non-randomized controlled trials (e.g., sequential trials, systematic reviews, case reports, clinical experiences, conference abstracts, animal studies, cellular studies) will not be considered.

#### 2.3.2 Types of participants

Due to the specific nature of ASD and its difficulties in early diagnosis,^[11]^ the age range of patients with ASD included in the study was 2 to 18 years, thus ranging from early childhood to adolescence. All participants, regardless of ethnic background and sex, were diagnosed with ASD according to relevant guidelines or consensus.

#### 2.3.3 Types of intervention

##### 2.3.3.1 Experimental groups

Due to ethical constraints, current research needs to be based on conventional interventions such as behavioral interventions that safeguard the basic rehabilitation rights of children with ASD without compromising them. Therefore, current clinical studies in ASD do not rely solely on TCM interventions, but are conducted in combination with behavioral intervention modalities. Based on the characteristics of TCM interventions for ASD and their applicability in clinical practice, we classified TCM interventions into 10 therapies^[12]^ (oral Chinese herbal medicine therapy, Chinese herbal infusion/fumigation therapy, Chinese herbal compress therapy, acupoint injection therapy, general acupuncture therapy, electro-acupuncture therapy, moxibustion therapy, tuina/massage/tactile stimulation therapy, cupping therapy, and Guasha therapy), which are detailed in Table 1.

**Table 1:** Detailed description of TCM interventions.

Intervention	Instruction
Oral Chinese herbal medicine therapy	It refers to the liquid preparation obtained by decocting herbs or coarse granules with water or boiling water and then removing the residue and extracting the liquid.
Chinese herbal infusion/fumigation therapy	A method of bathing the whole body or local area with herbal liquids or water containing herbal liquids.
Chinese herbal compress therapy	It is a treatment method of applying herbal preparations to the skin, orifices, acupuncture points, and localized lesions.
Acupoint injection therapy	It is a treatment method of injecting herbal liquid into acupuncture points to prevent and treat diseases.
General acupuncture therapy	Acupuncture is the stabbing of acupuncture points in the patient's body at a certain angle, thus achieving the purpose of treating the disease.
Electro-acupuncture therapy	A micro-current close to the body's bioelectricity is applied to the needles, using a combination of both needle and electrical stimulation.
Moxibustion therapy	The use of moxa or other drugs on the body surface of the acupuncture points burning, warm iron, through the heat of the moxibustion fire and the effect of drugs.
Tuina/massage/tactile stimulation therapy	Using manipulation techniques on specific parts of the body and acupuncture points.
Cupping therapy	It is a method of removing air from the tank by heat and using negative pressure to absorb it into the skin, causing the phenomenon of blood stasis.
Guasha therapy	Through the special scraping apparatus and corresponding techniques, dipping certain medium, repeatedly scraping and rubbing on the body surface to make the skin appear red corn-like locally.

The article "Traditional Chinese medicine intervention for autism spectrum disorders: A protocol for systematic review and network meta-analysis" was retracted in 2022. Reason: concerns about the citations.

##### 2.3.3.2 Control groups

The control group with non-TCM interventions will undergo only behavioral interventions or conventional intervention modalities.

#### 2.3.4 Types of outcomes

##### 2.3.4.1 Primary outcome(s)

The main efficacy evaluation index is based on the before-and-after results at the end of the intervention or at the end of the follow-up period to evaluate the effectiveness of the intervention. The efficacy, effectiveness, and ineffectiveness will be evaluated according to the relevant forms or questionnaires, which are based on research tools commonly used in clinical practice, including the ADOS (Autism Diagnostic Observation Scale), ADI-R (Autism Diagnostic Interview-Revised), and CARS (Childhood Autism Rating Scale). It is worth mentioning that even one of these questionnaires is sufficient for evaluation, considering their limited availability (in particular ADOS and ADI-R) in China due to copyright restrictions.

##### 2.3.4.2 Secondary outcomes

Secondary outcomes will include behavioral questionnaires, such as the autism behavior checklist and autism treatment evaluation checklist, to evaluate the effect of TCM on the improvement of ASD symptoms in multiple dimensions, and may also include some symptom score scales^[13]^

The article "Traditional Chinese medicine intervention for autism spectrum disorders: A protocol for systematic review and network meta-analysis" was retracted in 2022. Reason: concerns about the citations.

### 2.4 Database and search strategy

Starting in January 2022, we will conduct comprehensive searches in the following databases: China Biological Medicine Database, Chinese Scientific Journals Database, Wan Fang databases, China National Knowledge Infrastructure, the Cochrane Library, Web of Science, PubMed, and EMBASE Database. The language will be limited to English or Chinese, and our search formulae on PubMed are described in Table 2.

**Table 2:** PubMed search strategy protocol.

Number	Search items
#1	“Autism spectrum disorders”[Mesh]
#2	Autism[Title/Abstract] OR Autism Spectrum Disorders[Title/Abstract]
#3	#1 OR #2
#4	“Medicine, Chinese Traditional”[Mesh]
#5	“Acupuncture”[Mesh]
#6	“Electro-acupuncture”[Mesh]
#7	“Acupuncture Points”[Mesh]
#8	“Moxibustion”[Mesh]
#9	“Tuina”[Mesh]
#10	“Drugs, Chinese Herbal”[Mesh]
#11	“Cupping ”[Mesh]
#12	“Guasha ”[Mesh]
#13	Zhong Yi Xue[Title/Abstract] OR Medicine, East Asian Traditional[Title/Abstract] OR Acupuncture Therapy[Title/Abstract] OR Acupoint[Title/Abstract] OR trigger Points[Title/Abstract] OR Moxabustion[Title/Abstract] OR Massage[Title/Abstract] OR Tactile stimulation[Title/Abstract] OR Chinese Drugs, Plant[Title/Abstract] OR Herbal Drugs, Chinese[Title/Abstract] OR Plant Extracts, Chinese[Title/Abstract] OR Cupping Treatment[Title/Abstract] OR Acupoint sticking[Title/Abstract] OR Acupoint injection[Title/Abstract] OR Herb fumigation[Title/Abstract] OR Herb soaking[Title/Abstract] OR Scrapping[Title/Abstract]OR Chinese herbal infusiong [Title/Abstract]
#14	#4 OR #5 OR #6 OR #7 OR #8 OR #9 OR #10 OR #11 OR #12OR #13
#15	“Randomized Controlled Trial”[Publication Type]
#16	“Randomized Controlled Trials as Topic”[Mesh]
#17	“Pragmatic Clinical Trial”[Publication Type]
#18	“Pragmatic Clinical Trials as Topic”[Mesh]
#19	“Intention to Treat Analysis”[Mesh]
#20	“random allocation”[Mesh Terms]
#21	random∗[Title/Abstract]
#22	#14 OR #15 OR #16 OR #17 OR #18 OR #19 OR #20 OR #21
#23	#3 AND #13 AND #22

### 2.5 Literature selection and data extraction

First, the eligible literature will be imported into Endnote X8, and duplicate files will be removed. Next, two trained specialists (Xiang Feng and Keshang Li) will independently screen the eligible studies one by one based on the abstract and title, and studies that do not meet the inclusion criteria will be removed. In a second step full-text screening will be performed by the same two individuals, who will read each of the retrieved studies, and those that meet the criteria will be selected. In addition, the reasons for exclusion will be recorded. In the third step, the results will be cross-checked to ensure screening accuracy. When disagreement arises, a third senior assessor (Quanrui Jiang) will be consulted to reach consensus. The proposed flowchart is shown in Figure 1.

The article "Traditional Chinese medicine intervention for autism spectrum disorders: A protocol for systematic review and network meta-analysis" was retracted in 2022. Reason: concerns about the citations.

**Figure 1:** Flow chart of study selection.

After completing the above steps, a data extraction table will be created using Excel software as recommended in the Cochrane Handbook, which includes the name of the first author, year of publication, participant characteristics (sample size, sex, mean age, number of groups), interventions, comparative indicators, and outcomes. Since differences in baseline between samples can lead to differences in outcomes, in order to better assess the before and after changes in the efficacy of different TCM interventions for ASD, the final data included in the analysis will be calculated using the following formula from the Cochrane Handbook for Systematic Reviews of Interventions (version 5.1), where *r* is a correlation coefficient with a value of 0.5.^[14]^

### 2.6 Quality assessment

Quality assessment will be conducted by three researchers (Jun Yu, Yuxing Zhang, and Hui Zhi) to independently assess the risk of bias in all included randomized controlled trials using the Cochrane Collaboration tool, which focuses on the following aspects: task concealment, random sequence generation, blinding of outcome assessors, participant and personnel blinding, selective reporting, completeness of outcome data, and other sources of bias.^[15]^ Each domain was classified as high-risk, low-risk, or unclear risk. Should disagreements arise during the study, they will be resolved through discussion with a third senior assessor (Wu Li).

### 2.7 Statistical analysis

First, for the direct comparisons, a conventional meta-analysis will be performed using Revman 5.3 (Cochrane Collaboration, Oxford, UK). Second, considering the anticipated heterogeneity, the network meta-analysis within a Bayesian framework will be conducted using WinBUGS 1.4.3 (MRC Biostatistics Unit, Cambridge, UK) based on the random effect model for the results of the indirect comparison. In addition, models will be calculated using the Markov chain Monte Carlo algorithm^[16]^: four chains will be employed for simulation analysis, the step size will be set to 10, the number of annealing times will be set to 20,000 to reduce the impact on arbitrary values, and the number of iterations will be set to 50,000. Additionally, continuous outcomes will be measured by standard mean difference with 95% confidence intervals for indirect comparisons. Third, the plot of the surface under the cumulative ranking curve will be computed using STATA 14.0 (Stata Corporation, College Station, TX) to forecast the possible ranking order.^[17]^ In our study, a higher surface under the cumulative ranking curve score represents a better TCM intervention for ASD.^[12]^

The article "Traditional Chinese medicine intervention for autism spectrum disorders: A protocol for systematic review and network meta-analysis" was retracted in 2022. Reason: concerns about the citations.

### 2.8 Assessment of heterogeneity

We will assess whether participant characteristics, interventions, and outcomes are sufficiently similar across the included trials. If they are not, the heterogeneity of the outcomes will be assessed using *I* ^2^ in STATA 14.0. The software will only consider substantial heterogeneity if the *I* ^2^ value is above 50%, and a random effects model will be selected; otherwise, a fixed effects model will be used.

### 2.9 Assessment of inconsistency, subgroup, and sensitivity

In general, differences between different types of evidence may be the main reason for the inconsistency. Therefore, inconsistencies between indirect and direct evidence will be assessed using circular inconsistency tests and nodal splitting methods. In addition, *Z*-values and the corresponding *P*-values will be calculated, with *P*-values less than .05 indicating significant differences. If significant heterogeneity is found, subgroup analyses will be performed according to possible sources of heterogeneity, such as the severity of ASD in the children, age stratification, and evaluation forms.

### 2.10 Assessment of publication bias

To minimize the impact of study bias on the study results, we will adhere to the study principles outlined above. If sufficient studies are included (n > 10), we will use a funnel plot to assess bias.

### 2.11 Grading the quality of the evidence

The senior researcher (Jiangshan Li) will assess the quality of each article separately according to the GRADE working group methodology,^[18]^ which classifies the quality level into four categories: high, medium, low, and very low. Again, if there is uncertainty, a third-party evaluator will be consulted.

## 3 Conclusion

As a major neurodevelopmental disorder with no specific biological markers, ASD is extremely difficult to treat, and there is no specific treatment or intervention modality.^[19]^ Currently, global research on ASD focuses on its pathogenesis and clinical treatment. The use of interventional modalities in TCM has a positive impact on its efficacy. TCM interventions such as acupuncture^[20,21]^ and Tuina^[22,23]^ have been effectively used in the treatment of ASD. We believe that this systematic review and network meta-analysis will not only represent a substantial contribution to the recovery of patients but will also provide practitioners with clinical evidence to promote the use of TCM in ASD interventions.

The article "Traditional Chinese medicine intervention for autism spectrum disorders: A protocol for systematic review and network meta-analysis" was retracted in 2022. Reason: concerns about the citations.

## Acknowledgments

We are very grateful for the support of the teaching and research staff and graduate students of the Tuina Department of the School of Acupuncture and Tuina, Hunan University of Chinese Medicine.

## Author contributions

**Data curation:** Keshang Li, Quanrui Jiang, Yuxing Zhang, Zhichao Gong.

**Formal analysis:** Hui Zhi, Jun Yu.

**Funding acquisition:** Xiang Feng, Jiangshan Li.

**Investigation:** Keshang Li.

**Methodology:** Wu Li.

**Project administration:** Xiang Feng.

**Supervision:** Jiangshan Li.

**Writing – original draft:** Xiang Feng.

**Writing – review & editing:** Xiang Feng.
